# BCL6 Attenuates Proliferation and Oxidative Stress of Vascular Smooth Muscle Cells in Hypertension

**DOI:** 10.1155/2019/5018410

**Published:** 2019-01-22

**Authors:** Dan Chen, Ying-Hao Zang, Yun Qiu, Feng Zhang, Ai-Dong Chen, Jue-Jin Wang, Qi Chen, Yue-Hua Li, Yu-Ming Kang, Guo-Qing Zhu

**Affiliations:** ^1^Key Laboratory of Targeted Intervention of Cardiovascular Disease, Collaborative Innovation Center of Translational Medicine for Cardiovascular Disease, and Department of Physiology, Nanjing Medical University, Nanjing, Jiangsu 211166, China; ^2^Department of Pathophysiology, Nanjing Medical University, Nanjing, Jiangsu 211166, China; ^3^Department of Physiology and Pathophysiology, Cardiovascular Research Center, Xi'an Jiaotong University School of Medicine, Xi'an 710061, China

## Abstract

Proliferation and oxidative stress of vascular smooth muscle cells (VSMCs) contribute to vascular remodeling in hypertension and several major vascular diseases. B-cell lymphoma 6 (BCL6) functions as a transcriptional repressor. The present study is designed to determine the roles of BCL6 in VSMC proliferation and oxidative stress and underlying mechanism. Angiotensin (Ang) II was used to induce VSMC proliferation and oxidative stress in human VSMCs. Effects of BCL6 overexpression and knockdown were, respectively, investigated in Ang II-treated human VSMCs. Therapeutical effects of BCL6 overexpression on vascular remodeling, oxidative stress, and proliferation were determined in the aorta of spontaneously hypertensive rats (SHR). Ang II reduced BCL6 expression in human VSMCs. BCL6 overexpression attenuated while BCL6 knockdown enhanced the Ang II-induced upregulation of NADPH oxidase 4 (NOX4), production of reactive oxygen species (ROS), and proliferation of VSMCs. BCL6 expression was downregulated in SHR. BCL6 overexpression in SHR reduced NOX4 expression, ROS production, and proliferation of the aortic media of SHR. Moreover, BCL6 overexpression attenuated vascular remodeling and hypertension in SHR. However, BCL6 overexpression had no significant effects on NOX2 expression in human VSMCs or in SHR. We conclude that BCL6 attenuates proliferation and oxidative stress of VSMCs in hypertension.

## 1. Introduction

Vascular smooth muscle cells (VSMCs) are dominant cellular constituent of arteries [1, 2]. VSMC proliferation is closely linked with vascular remodeling and stiffening in the initiation and progression of vascular diseases such as hypertension, atherosclerosis, myocardial hypertrophy, myocardial infarction, stroke, dementia, and renal failure [3–5]. Nicotinamide adenine dinucleotide phosphate (NADPH) oxidase (NOX) is a major source of reactive oxygen species (ROS) in VSMCs and is essential to cell proliferation [6]. It is known that Ang II binds to Ang II type 1 receptor (AT_1_R) and consequently activates NOX and promotes ROS generation and VSMC proliferation [7–9]. Angiotensin II (Ang II) is associated with the pathogeneses of hypertension and cardiovascular remodeling [10–12]. Intervention of renin-angiotensin system in hypertensive patients lowers morbidity and mortality [13, 14].

B-cell lymphoma 6 (BCL6) is initially discovered as an oncogene in B-cell lymphomas. It drives the malignant phenotype by repressing proliferation and DNA damage checkpoints and blocking B-cell terminal differentiation, and BCL6 inhibitors yield dramatic antitumor effects [15]. BCL6 protein is an evolutionarily conserved zinc finger transcription factor with an N-terminal POZ/BTB domain. This protein interacts with several corepressor complexes to inhibit transcription and functions as a sequence-specific transcriptional repressor [16]. BCL6 member B (BCL6B), a BCL6 homologous gene, suppresses proliferation of colorectal carcinoma cells through inhibition of the PI3K signaling pathway [17]. BCL6 is considered as a therapeutic target for autoimmune diseases and cancer treatment [15]. BCL6 overexpression inhibits ROS generation and apoptosis induced by chemotherapy in B-cell lymphoma cells [18]. However, it is unknown whether BCL6 plays a role in vascular remodeling in hypertension. This study reveals the role of BCL6 in inhibiting Ang II-induced VSMC proliferation and oxidative stress and attenuating vascular remodeling in hypertensive rats.

## 2. Materials and Methods

### 2.1. Animals

Thirteen-week-old male spontaneously hypertensive rats (SHR) and Wistar-Kyoto rats (WKY) were obtained from Vital River Laboratory Animal Technology Co. Ltd. (Beijing, China) and housed in a temperature-controlled room with a 12 h light/dark cycle and free access to standard chow and tap water. Experiments were approved by the Experimental Animal Care and Use Committee of Nanjing Medical University and the Guide for the Care and Use of Laboratory Animal published by the US National Institutes of Health (NIH publication, 8th edition, 2011). At the end of experiments, each rat was euthanized with an overdose of pentobarbital sodium (150 mg/kg, iv), and the aorta was harvested for histological and molecular biological analyses.

### 2.2. Cell Culture

Human aortic VSMCs were obtained from the American Type Culture Collection (Rockville, MD, USA) and cultured as described previously [3]. Simply, the VSMCs were cultured in F12K Kaighn's modification medium supplemented with 10% fetal bovine serum (FBS), 100 units/mL penicillin, and 100 mg/mL streptomycin at 37°C in a humidified atmosphere containing 5% CO_2_. The medium was replaced at intervals of 3-4 days. The cells were starved for 24 h in a serum-free medium before use [19].

### 2.3. BCL6 Overexpression in VSMCs

BCL6 overexpression plasmid was constructed by Hanbio Biotechnology Co. Ltd. (Shanghai, China) as reported previously [20]. Simply, BCL6-gene cDNA cloned by PCR was inserted into CMV-MCS-T2A-EGFP vectors, and the plasmid was verified by sequencing. VSMCs were seeded in 6-well plates at a density of 1 × 10^5^ cells/mL. After 80% confluent, the cells were transfected with pcDNA3.1 plasmid (control) or BCL6 overexpression plasmid (1 *μ*g/mL) using Lipofectamine 3000 for 24 h. Then, the transfected VSMCs were treated with PBS or Ang II (100 nM) for 48 h.

### 2.4. BCL6 Knockdown in VSMCs

BCL6 knockdown was carried with BCL6 short-hairpin RNA (shRNA) in VSMCs, which were constructed by GeneChem (Shanghai, China) as reported previously [20]. The sequence used in the present study was 5′-AGTGAAGCAGAGATGGTTT-3′ for BCL6 shRNA and 5′-TTCTCCGAACGTGTCACGT-3′ for scramble-shRNA (control). VSMCs were treated with Scr-shRNA or BCL6 shRNA (1 *μ*g/mL) for 24 h followed by treatment with PBS or Ang II (100 nM) for 48 h.

### 2.5. BCL6 Overexpression in WKY and SHR

BCL6 overexpression lentivirus vector and enhanced red fluorescent protein (ERFP) lentivirus vector were constructed by Obio Technology Corp., Ltd. (Shanghai, China) [20]. WKY and SHR aged 13 weeks were subjected to intravenous injection of recombinant lentivirus expressing BCL6 or ERFP (2 × 10^9^ TU/mL, 50 *μ*L). Acute experiments were carried out 4 weeks after the lentivirus induction.

### 2.6. CCK-8 Assay

Cell counting kit-8 kits (CCK-8, Beyotime Institute of Biotechnology, Shanghai, China) were used for evaluating VSMC proliferation according to the manufacturer's instructions. As we reported previously [3], 10 *μ*L of CCK-8 solution was added into each well and incubated for 2 h at 37°C. The absorbance was measured at 450 nm with a microplate reader (ELX800, BioTek, Vermont, USA).

### 2.7. EdU Incorporation Assay

EdU incorporation assay was used to determine VSMC proliferation with In Vitro Imaging Kit (Guangzhou RiboBio, Guangzhou, China). The DNA synthesis of VSMCs was measured using a Cell-Light™ EdU Apollo®567. The EdU-positive cells were counted and normalized by the total number of Hoechst 33342 stained cells [3].

### 2.8. RT-PCR

Total RNA was isolated with Trizol reagent (Life Technologies, Gaithersburg, MD, USA) according to the manufacturer's instruction. Reverse transcriptase reactions were performed using the PrimeScript RT reagent Kits. RT-PCR was performed using Quantitative PCR with SYBR Premix Ex Taq TM (Takara, Otsu, Shiga, Japan) and ABI PRISM 7500 sequence detection PCR system (Applied Biosystems, Foster City, CA, USA). The expressions of mRNA were calculated using the comparative cycle threshold (Ct) method where the relative quantization of target transcript levels was determined by subtracting Ct values of target genes from Ct values of GAPDH. The sequences of primers for humans and rats were listed in Tables 1 and 2.

### 2.9. Western Blot Analysis

Samples were homogenized in a lysis buffer. A protein assay kit (BCA; Pierce, Santa Cruz, CA, USA) was used for the measurement of total protein in the supernatant. Total protein was separated in SDS-PAGE and transferred to PVDF membranes in Tris-glycine-methanol buffer. The bands were visualized using enhanced chemiluminescence. GADPH was used as a loading control to normalize the data. Rabbit monoclonal antibody against BCL6 (1 : 1000) was purchased from Cell Signaling Technology (Beverly, MA, USA). Rabbit polyclonal antibodies against PCNA (1 : 1000), NOX2 (1 : 1000), and NOX4 (1 : 1000) were obtained from Proteintech Group (Wuhan, Hubei, China). Mouse monoclonal antibody against GAPDH (1 : 800) was obtained from Santa Cruz Biotechnology (Santa Cruz, CA, USA).

### 2.10. DHE Fluorescence Staining

Intracellular ROS in VSMCs or aorta were evaluated with dihydroethidium (DHE) staining. Cells (3 × 10^5^ cells/mL) in six-well plates were incubated with DHE (10 *μ*M) in PBS for 30 min in a dark and humidified container at 37°C and then washed twice with cold PBS. Sections of OCT-embedded aorta tissues were incubated with the same concentration of DHE for 5 min at room temperature and rinsed two times with PBS. The fluorescence signals were obtained with a fluorescence microscopy under excitation at 518 nm and emission at 605 nm (DP70, Olympus Optical, Tokyo, Japan).

### 2.11. Measurement of NAD(P)H Oxidase Activity

NAD(P)H oxidase activity was measured with enhanced lucigenin chemiluminescence method as we previously reported [21]. Homogenate supernatant of the sample was diluted in a modified HEPES buffer with SOD (350 U/mL). NAD(P)H (100 *μ*M) was used as a substrate for generating superoxide anions in the reaction system. The reaction between superoxide anions and lucigenin started at the time of adding dark-adapted lucigenin (5 *μ*M). Light emission was measured for 10 times in 10 min with a luminometer (20/20n, Turner, CA, USA). The values were expressed as RLU per minute per milligram of protein.

### 2.12. Statistical Analysis

Two-way ANOVA followed by post hoc Bonferroni test was used for multiple comparisons. All data were expressed as mean ± SE. A value of *P* < 0.05 was considered statistically significant.

## 3. Results

### 3.1. BCL6 Overexpression Inhibits Ang II-Induced VSMC Proliferation

VSMC proliferation was evaluated with CCK-8 kit, EdU assay, and proliferating cell nuclear antigen (PCNA) expression. CCK-8 assay showed that Ang II-induced VSMC proliferation was inhibited by BCL6 overexpression (Figure 1(a)). EdU incorporation assay detects DNA synthesis in proliferating cells. BCL6 overexpression inhibited the increase in the number of EdU-positive cells caused by Ang II in VSMCs (Figures 1(b) and 1(c)). PCNA is an essential component at the DNA replication and a key marker involved in DNA replication and cell proliferation. Ang II increased PCNA expression in VSMCs, which was attenuated by BCL6 overexpression (Figure 1(d)). On the other hand, Ang II reduced BCL6 expression in VSMCs. The effectiveness of the BCL6 overexpression was confirmed by the increased BCL6 protein level in VSMCs (Figure 1(e)).

### 3.2. BCL6 Overexpression Attenuates Ang II-Induced Oxidative Stress in VSMCs

Ang II increased NOX2 and NOX4 mRNA levels in VSMCs. BCL6 overexpression significantly reduced NOX4 mRNA expression rather than NOX2 mRNA expression (Figure 2(a)). Similarly, BCL6 overexpression inhibited Ang II-induced upregulation of NOX4 protein expression rather than NOX2 protein expression (Figure 2(b)). Ang II increased NAD(P)H oxidase activity, which was inhibited by BCL6 overexpression (Figure 2(c)). Dihydroethidium (DHE) staining showed that ROS production was increased in Ang II-treated VSMCs, which was attenuated by the BCL6 overexpression (Figures 2(d) and 2(e)).

### 3.3. BCL6 Knockdown Intensified Effects of Ang II in VSMCs

Knockdown of BCL6 with shRNA in VSMCs aggravated Ang II-induced VSMC proliferation evidenced by the increased absorbance measured with CCK-8 assay (Figure 3(a)) and the upregulation of PCNA protein expression (Figure 3(b)). BCL6 knockdown had no significant effect on NOX2 protein expression but aggravated Ang II-induced upregulation of NOX4 protein in VSMCs (Figure 3)(c). Moreover, Ang II-induced ROS production was increased by BCL6 knockdown (Figures 3(d) and 3(e)). The effectiveness of BCL6 knockdown was confirmed by the downregulation of BCL6 protein in VSMCs (Figure 3(f)).

### 3.4. BCL6 Overexpression Attenuates Vascular Remodeling in SHR

Recombinant lentivirus expressing BCL6 was administrated intravenously to induce BCL6 overexpression in WKY and SHR. The effectiveness of BCL6 overexpression was confirmed by the upregulation of BCL6 protein expression in the aortic media of both WKY and SHR. Moreover, the BCL6 protein expression in the aortic media was downregulated in SHR (Figure 4(a)). BCL6 overexpression attenuated the upregulation of PCNA protein expression in the aortic media of SHR (Figure 4(b)). Masson's staining showed that BCL6 overexpression attenuated vascular remodeling in SHR (Figure 4(c)). Media thickness (M), lumen diameter (L), and their ratio of artery were used as indexes of vascular remodeling [22]. Increased M and M/L in the aorta of SHR were prevented by BCL6 overexpression (Figure 4(d)). In addition, BCL6 overexpression reduced systolic blood pressure (SBP) and mean arterial pressure (MAP) in SHR (Figure 4(e)).

### 3.5. BCL6 Overexpression Attenuates Oxidative Stress in the Aorta of SHR

Both NOX2 and NOX4 mRNA and protein expressions in the aortic media were increased in SHR compared with those in WKY. BCL6 overexpression attenuated the NOX4 mRNA and protein upregulation in SHR rather than the NOX2 mRNA and protein upregulation (Figures 5(a) and 5(b)). DHE staining revealed that the ROS level in the aorta was greatly increased in SHR, which was attenuated by BCL6 overexpression (Figures 5(c) and 5(d)).

## 4. Discussion

VSMC proliferation contributes to vascular remodeling in several major vascular diseases including hypertension, pulmonary arterial hypertension, atherosclerosis, vascular restenosis, transplantation arteriopathy, and diabetic vascular complications [2]. Oxidative stress is a critical factor in promoting cell proliferation [23]. Primary novel findings in the present study are that BCL6 inhibits Ang II-induced oxidative stress and proliferation in human VSMCs, and BCL6 overexpression attenuates oxidative stress and vascular remodeling in the aorta of SHR. BCL6 reduces NOX4 expression, which may contribute to its antioxidative effect in Ang II-treated VSMCs or the aorta of SHR.

Ang II plays a crucial role in hypertension and its associated organ damage [14]. Blockade of AT_1_R or inhibition of Ang II generation is an important strategy for the treatment of hypertension [13]. Ang II is widely used to induce hypertension and vascular remodeling as an animal model of hypertension [24–26]. It is well known that Ang II induces VSMC proliferation [27], which is widely used as a model of VSMC proliferation *in vitro* [28–30]. We found that BCL6 overexpression attenuated while BCL6 knockdown enhanced the Ang II-induced VSMC proliferation, indicating that BCL6 is an important protective factor in inhibiting Ang II-induced VSMC proliferation. More importantly, BCL6 overexpression in SHR attenuated vascular remodeling and reduced PCNA expression in the aortic media of SHR. The *in vivo* study provides evidence that BCL6 is important in attenuating vascular remodeling and VSMC proliferation in SHR. The inhibitory effect of BCL6 on VSMC proliferation at least partially contributed to its role in attenuating vascular remodeling in SHR.

It is noted that Ang II reduced BCL6 expression in human VSMCs, and BCL6 expression was downregulated in the aortic media of SHR, suggesting that the reduced BCL6 levels may be involved in the enhanced VSMC proliferation in both Ang II-treated VSMCs and aortic media of SHR. However, the mechanisms of the BCL6 downregulation are not known, which need further investigation. On the other hand, BCL6 overexpression had no significant effect on blood pressure in normotensive WKY but reduced blood pressure in SHR. The attenuated vascular remodeling caused by BCL6 in hypertension may partially contributes to its antihypertensive effect. We recently have shown that BCL6 attenuates renal inflammation via negative regulation of NLRP3 transcription in SHR, which may be also involved in its antihypertension effect [20].

Oxidative stress is associated with vascular defects leading to hypertension and atherosclerosis [31, 32]. Removal of excess ROS is a therapeutic strategy for oxidative stress-related cardiovascular diseases [33–35]. Accumulating evidences have shown that Ang II activates NOXs mediated by AT_1_R, which promotes ROS generation and subsequent VSMC proliferation [7–9]. BCL6 knockdown increased the transcription of NADPH oxidase subunits P67 and gp91 in normal cardiomyocytes, and hypoxia-induced P67 and gp91 upregulation in cardiomyocytes was enhanced by Bcl6 knockdown [36]. We found that Ang II-induced NAD(P)H oxidase activation, ROS generation, and NOX4 upregulation were attenuated by BCL6 overexpression but exacerbated by BCL6 knockdown in human VSMCs. However, Ang II-induced NOX2 upregulation was not significantly affected by BCL6 overexpression or knockdown. The findings were supported by the *in vivo* study that BCL6 overexpression in SHR attenuated the increased ROS production and NOX4 upregulation but had no significant effect on the NOX2 upregulation in the aortic media of SHR. These results indicate that BCL6 attenuates oxidative stress in Ang II-treated VSMCs and aortic media of SHR, which may be related to the downregulation of NOX4. The antioxidative effects of BCL6 in VSMCs were supported by previous findings that BCL6 overexpression inhibited oxidative stress response to etoposide and other chemotherapeutic reagents in B-cell lymphoma cells [18] and that BCL6 knockdown augmented the hypoxia-induced oxidative stress in cardiomyocytes [36]. The limitations in the present study were that the effect of specific inhibitor of NOX-2 or NOX-4 on DHE staining was not examined and that DHE staining was used to evaluate ROS production for in vivo experiments instead of a widely accepted marker of oxidative stress.

In summary, BCL6 is downregulated in Ang II-treated human VSMCs and aortic media of SHR. BCL6 overexpression attenuates while BCL6 knockdown exacerbates Ang II-induced oxidative stress and proliferation of human VSMCs. BCL6 overexpression inhibits oxidative stress and proliferation of aortic media in SHR. BCL6 inhibits NOX4 expression, which may contribute to its antioxidative effect in Ang II-treated VSMCs and in the aortic media of SHR.

## Figures and Tables

**Figure 1:** Effects of BCL6 overexpression (OE) on Ang II-induced VSMC proliferation. VSMCs were treated with empty plasmid or BCL6 plasmid (1 *μ*g/mL) for 24 h followed by PBS or Ang II (100 nM) treatment for 48 h. (a) VSMC proliferation was determined with CCK-8 assay. *n* = 6. (b) Percentage of EdU-positive cells. (c) Representative images showing EdU-positive cells measured with Edu incorporation assay. Blue fluorescence shows cell nuclei and red fluorescence stands for cells with DNA synthesis. (d) PCNA protein expression. (e) BCL6 protein expression. Values are mean ± SE. ^∗^*P* < 0.05 vs. PBS; †*P* < 0.05 vs. Ctrl. *n* = 6 in (a) and (b); *n* = 4 in (c) and (d).

**Figure 2:** Effects of BCL6 overexpression (OE) on Ang II-induced oxidative stress in VSMCs. The VSMCs were treated with empty plasmid or BCL6 plasmid (1 *μ*g/mL) for 24 h followed by PBS or Ang II (100 nM) treatment for 48 h. (a) NOX2 and NOX4 mRNA levels. (b) NOX2 and NOX4 protein expressions. (c) NAD(P)H oxidase activity. (d) ROS detected by dihydroethidium (DHE) staining. (e) Bar graph showing the relative fluorescence intensity of DHE. Values are mean ± SE. ^∗^*P* < 0.05 vs. PBS; †*P* < 0.05 vs. Ctrl. *n* = 4 in (a) and (b); *n* = 6 in (c) and (d).

**Figure 3:** Effects of BCL6 knockdown on Ang II-induced VSMC proliferation and oxidative stress in VSMCs. The cells were treated with Scr-shRNA or BCL6 shRNA (1 *μ*g/mL) for 24 h followed by treatment with PBS or Ang II (100 nM) for 48 h. (a) VSMC proliferation determined by CCK-8 assay. (b) PCNA protein expression. (c) NOX2 and NOX4 protein expressions. (d) ROS detected by dihydroethidium (DHE) staining. (e) Bar graph showing the relative fluorescence intensity of DHE. (f) BCL6 protein expression. Values are mean ± SE. ^∗^*P* < 0.05 vs. PBS; †*P* < 0.05 vs. Ctrl. *n* = 6 for each group.

**Figure 4:** Effects of BCL6 overexpression (OE) on vascular remodeling of aorta and blood pressure in WKY and SHR. (a) BCL6 protein expression in media of aorta. (b) PCNA protein expression in media of aorta. (c) Representative transverse section images of aorta with Masson's stain. (d) Bar graph showing the media thickness (M), lumen diameter (L), and the ratio of M to L. (e) Systolic blood pressure (SBP), mean arterial pressure (MAP), and heart rate (HR). Values are mean ± SE. ^∗^*P* < 0.05 vs. WKY; †*P* < 0.05 vs. Ctrl. *n* = 6 for each group.

**Figure 5:** Effects of BCL6 overexpression (OE) on oxidative stress in the aortic media of WKY and SHR. (a) NOX2 and NOX4 mRNA levels. (b) NOX2 and NOX4 protein expressions. (c) ROS detected by dihydroethidium (DHE) staining in aorta. (d) Bar graph showing the relative fluorescence intensity of DHE. Values are mean ± SE. ^∗^*P* < 0.05 vs. WKY; †*P* < 0.05 vs. Ctrl. *n* = 6 for each group.

**Table 1:** Primers for real-time quantitative PCR analysis in humans.

	Primer	Sequence
NOX2	Forward	GAGTTGTCATCACGCTGTGC
	Reverse	CCACGTACAATTCGTTCAGC
NOX4	Forward	ACAACTGTTCCTGGCCTGAC
	Reverse	CGGGAGGGTGGGTATCTAAA
GAPDH	Forward	AACAGCGACACCCACTCCTC
	Reverse	GGAGGGGAGATTCAGTGTG

**Table 2:** Primers for real-time quantitative PCR analysis in rats.

	Primer	Sequence
NOX2	Forward	ACCAAGGTGGTCACTCATCC
	Reverse	ACAATGCGGATATGGATGCT
NOX4	Forward	ACAGTCCTGGCTTACCTTCG
	Reverse	CTGAGAAGTTCAGGGCGTTC
GAPDH	Forward	TGAGGCCGGTGCTGAGTATGT
	Reverse	CAGTCTTCTGGGTGGCAGTGAT

## Data Availability

The data used to support the findings of this study are available from the corresponding author upon request.
